The article "Construction and Simulation of Financial Audit Model Based on Convolutional Neural Network" was retracted in 2023. Reasons: unreliable results or conclusions; concerns about the data; concerns about the results or conclusions; concerns about the peer review.

# Construction and Simulation of Financial Audit Model Based on Convolutional Neural Network

**DOI:** 10.1155/2021/1182557

**Published:** 2021-07-01

**Authors:** Xiaoyi Zhang

**Affiliations:** School of Accounting, Tongling University, Tongling, Anhui 244061, China

## Abstract

Big data has brought a new round of information revolution. Faced with the goal of full coverage of audit and supervision, making full use of big data is the main method to promote the realization of the goal of full coverage of audit and supervision. Data analysis and utilization is an indispensable task of auditing. Actively exploring multidimensional and intelligent data analysis methods and developing big data audit cases are the new development direction of auditing. The convolutional neural network's excellent ability to extract data features well meets the relevant requirements of financial auditing. However, in practical applications, convolutional neural networks often encounter various problems such as disappearance of gradients and difficulty in convergence, which reduces its expected performance in financial audit applications. In order to make the performance of the financial audit model based on convolutional neural network more excellent, after summarizing the characteristics of genetic algorithm, this article applies genetic algorithm to the optimization of the convolutional neural network model. We applied genetic algorithm to optimize the initial weights of the convolutional neural network. The error sensitivity and learning rate changes of different hidden layers are discussed, the influence of different learning rates on the convergence speed of convolutional neural networks is analyzed, and the recognition performance of other algorithms on financial audit data sets is simulated and compared. We conducted experiments on the network structure and parameter optimization on the financial audit database. The results show that the recognition error rate of the convolutional neural network model with improved learning rate algorithm in the financial audit data set is lower than that of the multilayer feedforward network, so it has better performance.

## 1. Introduction

With its globalization characteristics, the development of the financial industry in the 21st century not only shows globalization and informatization, but also is developing towards “cloud.” With the continuous deepening of the reform of the domestic financial industry, the mixed operation of the financial industry has become more and more obvious, which has led to changes in the financial auditing information environment [1, 2]. In the modern national economic system, finance is at the core. When “cloud computing” is widely integrated into our modern information life, if auditors can design and innovate audit methods and technologies from the perspective of “cloud computing,” they can deal with the intricate financial “cloud” environment and establish a sound financial supervision system [3].

In the environment of the big data era, the global financial industry is experiencing an information revolution of “data cloudification, information cloudification.” Computer-based intelligent cloud-based tools are gradually changing the working methods and transaction patterns of financial practitioners [4]. As many government financial institutions have taken the lead in implementing electronic and networked management, and the characteristics of complex and diversified data, government financial auditing should also move towards the construction of cloud-based auditing in the same way as the development of the financial industry, so as to achieve cloud-based auditing and supervision [5]. For electronic financial data at the information level, the use of big data ideas to design new audit methods is of great significance for achieving audit goals and creating a new model of auditing “clouds” [6].

This article briefly describes the concept of data mining and exemplifies the methods that may be used in financial audit data mining. It also sorts out the main methods of financial audit in detail and describes its business content, audit ideas, and how to use data mining methods to achieve audit based on these methods. This paper analyzes the convolutional neural network in detail, introduces the related ideas of genetic algorithm, and describes the process and application of genetic algorithm in detail. According to the problems in the training process of convolutional neural network, genetic algorithm is applied to the parameter optimization of convolutional neural network, and the specific optimization process of this method is given. This paper studies the gradient of different hidden layers with Min batch, analyzes the impact of different learning rates on network accuracy and convergence, and focuses on the impact of increasing the weight term (L1) regularization method on the network generalization ability. We designed three sets of parameter models for comparative analysis and finally selected a model with a weight attenuation coefficient of 5. The stochastic gradient descent algorithm of the improved learning rate algorithm is used to train parameters on the MNISI data set, and the influence of the relevant parameters of the model on the recognition rate is analyzed through experiments, and the error rate of other algorithms is compared to verify the feasibility of the algorithm.

## 2. Background and Related Works

Data mining, also known as knowledge discovery, refers to the process of discovering interesting and potentially useful information from large-scale data, as well as the potential, inherent, and useful patterns or models of the data itself. Data mining is not an independent discipline. It integrates the relevant theories and technologies of statistics, computer science, artificial intelligence, pattern recognition, database and other disciplines, and its application models are diverse, mainly including classification models, prediction models, cluster analysis and association rule analysis, etc. With the increasing and frequent financial activities, financial data also grows rapidly, and it is no longer possible to process a large amount of financial data only by relying on human resources [7, 8]. Therefore, data mining methods have also become commonly used methods in the financial forecasting field. At present, data mining technology has been widely used in financial forecasting fields such as stocks, bankruptcy assessment, exchange rates, and futures. Using data mining methods can dig out hidden laws or patterns from existing financial data without requiring any assumptions or fewer assumptions, and use these laws or patterns to predict future trends in financial activities. Data mining methods currently used in the field of financial forecasting mainly include artificial neural networks, support vector machines, genetic algorithms, and hidden Markov models [9–11].

Neural network is a method of learning from training samples and obtaining the mapping relationship from input to output through the calculation of a large number of connected neurons. Relevant scholars have proposed a financial forecasting model based on the generalized regression neural network method, which can increase the calculation speed, and at the same time, the forecasting performance is better than the traditional BP neural network [12–14]. The BP neural network prediction model can effectively capture the nonlinear characteristics in the data and is suitable for binary, multivariate, and continuous data. However, the setting of network parameters will affect the prediction effect. If the training process is not properly controlled or parameter settings are set, it is easy to overfit. Genetic algorithm is a combinatorial optimization algorithm that uses the evolutionary principles of natural selection and survival of the fittest. The basic principle is that given an objective function, by inheriting and mutating the genetic code, the fitness of the candidate solution is continuously improved until the optimal solution is found [15, 16].

Related scholars have successfully applied neural networks to short-term stock index forecasts, and related researchers have continuously proposed various types of neural network structures and applied them in financial forecasts [17–19]. Researchers used an adaptive BP neural network to predict the changing trends of two important stock indexes, S&P500 and NIKKEI225, and achieved good results [20, 21]. Researchers combined knowledge discovery (MMDR) with neural networks and achieved prediction results superior to traditional methods [22–24]. Relevant scholars combined genetic algorithm with ARIMA model, optimized the coefficients of ARIMA model through genetic algorithm, and improved the prediction accuracy [25]. Researchers proposed that combining multiple population genetic algorithms with neural networks can consider both global and local optimization solutions [26]. Genetic algorithm can be used to solve high-dimensional and non-linear problems, but due to the limitations of the coding mechanism, it will be difficult or too long to encode continuous variables. The support vector machine is essentially a binary classification model that takes the structural risk minimization as the criterion and maximizes the classification hyperplane interval of the feature space as the optimal goal. It learns through training samples to find the classification hyperplane with the largest interval, that is, the optimal classification hyperplane, and uses the hyperplane as a decision-making surface to realize functions such as classification, prediction, or regression.

Relevant scholars pointed out that it is necessary to clarify the positioning and objectives of financial auditing, grasp the key points and main lines of financial auditing, and innovate auditing methods to face the opportunities and challenges brought about by economic globalization [27, 28]. In the context of the financial crisis, researchers pointed out that there are many contradictions in financial auditing [29]. In order to resolve the contradictions, a coordination mechanism between financial auditing and financial supervision should be established, making full use of financial risk management techniques, enhancing the data processing capabilities of audit workers, and giving full play to auditing. Relevant scholars also believe that financial auditing should give full play to its unique advantages of independence, work with financial regulatory agencies to play a re-supervision function, and jointly maintain national financial security by strengthening the mutual cooperation between government financial auditing agencies and national financial regulatory agencies [30].

After data collection, audit institutions at all levels required the construction of a new data service center. On the premise of ensuring data security, they standardize the scope of authority for auditors to retrieve data, provide data import, cleanup, analysis, and output, and serve the development of audit projects [31]. At present, audit institutions at all levels have at least one computer auditing talent who has passed intermediate training in computer auditing [32]. Through these computer auditing talents, they can play their seed role in the unit and establish a special computer research team or data analysis room to manage data and explore the value of data in depth. Relevant departments have invited audit backbones from different business offices to participate in the data mining work and establish a cross-professional audit data mining research team [33].

## 3. Key Technologies of Financial Audit Data Mining

### 3.1. Data Mining Technology

Data mining is the process of extracting potentially useful information and knowledge hidden in it from a large amount of incomplete, noisy, fuzzy, and random practical application data. Data mining modes can often be divided into two types: one is supervised data mining, and the other is unsupervised data mining. Supervised data mining is that mining personnel have clear needs and goals. For financial audits, this mining mode can be used to collect basic financial information. Unsupervised data mining uses a certain method to find regularities or abnormalities in the data and submit them to the user, and the user judges the degree of importance. For financial auditing, this mining mode can be used to find problems, and it is a common data mining method for auditors. The financial audit platform based on big data is shown in Figure 1.

Data mining can be performed on a wide range of data objects. It can mine structured data generated by information system databases, as well as semi-structured data such as graphics, text, and images. The basic algorithms of data mining include classification mining method, association mining method, cluster mining method, and heterogeneous mining method. In financial auditing, the above-mentioned data mining algorithms can be modeled and then solidified, and the required models can be selected and applied according to the characteristics of the data and audit objectives. When financial auditing analyzes the basic situation of fiscal operation, if you choose classification and other models for forecasting, combine the macro data such as GDP, CPI, power consumption, corporate energy consumption, and other data with fiscal budget revenue, fiscal budget expenditure, and other data for data; comprehensive analysis can analyze and evaluate the degree of achievement of macro policy objectives, and provide decision-making support for the implementation and improvement of fiscal policies. When auditing the allocation and management of fiscal funds, association analysis and cluster analysis models can be used to find loopholes or deficiencies in the funds management mechanism of the financial sector, promote the scientific standardization of fiscal management, and improve the use of fiscal funds. In the standard audit of fiscal internal control procedures, anomaly detection models can be used to find false information and deliberate behavior in fiscal funds payments; when methods such as decision numbers are used, the accuracy and efficiency of dynamic monitoring of fiscal funds receipts and payments can be improved.

Classification technology is an important part of data mining. The methods that can be applied to financial auditing are as follows:

1. *Decision Tree Algorithm*. Decision tree algorithm is currently one of the most widely used inductive reasoning algorithms. It is an algorithm that approximates discrete value function data, and it should be regarded as a “Boolean function.” This algorithm is an example-based learning algorithm, usually used to form classifiers and prediction models, focusing on inferring classification rules in the form of decision-making over several years from a set of disorderly and irregular examples.
2. *Bayesian Algorithm*. Bayesian algorithm is a statistical algorithm based on Bayes' theorem. The algorithm can estimate the possibility of class membership, such as the probability that a given sample belongs to a particular class, and get the classification of a given sample.
3. *Artificial Neural Network*. Artificial neural network is the most important tool in classification technology. It can be divided into four types: forward type, feedback type, stochastic type, and self-organizing competition type. It is a nonlinear model that allows it to flexibly simulate real-world data.

### 3.2. Financial Audit Methods

Financial audit methods are applied to financial business touch points such as fiscal budget and final accounts audit, department budget and final accounts audit, tax audit, financial audit, social security audit, etc., and also include various key links, such as non-tax revenue collection and management, and bank entity accounts. Special audits such as management and “three public funds” have strong practicability.

The General Office of the National Audit Office divides the audit matters of financial audit into three parts: budget execution audit, department budget execution audit, and financial special audit. Each business includes several audit items. Based on the summary of financial auditing practices over the years, the audit methods that can be applied to financial auditing data mining mainly include the following:

1. Budget implementation progress audit method: government budget implementation progress forecast, fiscal special fund budget implementation progress forecast, department budget implementation progress forecast; government budget implementation progress warning, financial special fund budget implementation progress warning, department budget implementation progress.
2. Fiscal revenue analysis and audit methods: the authenticity of fiscal revenue; the quality of fiscal revenue; the compliance of fiscal revenue collection; the rationality of fiscal revenue matching.
3. Index management and distribution audit methods: general index detail inquiry, department index detail inquiry, unit index detail inquiry, overall index execution inquiry, department index execution inquiry, and unit index execution inquiry.
4. Financial payment management audit methods: analysis of the proportion of direct fiscal payment and authorized payment, analysis of the proportion of fiscal funds allocated to the central treasury payment, analysis of the use of official business cards, analysis of large-value payments, transfer of state treasury funds to entity accounts, personal analysis of the payee, etc.
5. Other audit methods: consistency analysis of fiscal revenue accounts, comparison analysis of fiscal revenue budget and final accounts, consistency analysis of fiscal expenditure accounts, comparison analysis of fiscal expenditure budget and final accounts, analysis of non-tax revenue bills, and government procurement over-budget expenditure query and other audit methods.

## 4. Financial Audit Model of Convolutional Neural Network Improved Based on Genetic Algorithm

### 4.1. Analysis of Convolutional Neural Network Structure

Convolutional neural networks can extract the features of the data layer by layer to learn more refined features. Generally speaking, the feature extraction stage is completed by a convolutional layer and a pooling layer. The convolutional neural network is composed of multiple convolutional layers and pooling layers. The classifier can be composed of a multi-layer neural network.  Figure 2 shows the structure of a convolutional neural network [34].

The convolutional layer is the core of the convolutional neural network. The neurons of the convolutional layer will extract the features of the corresponding part of the area in the feature map of the previous layer. The input feature map and the 3 × 3 convolution kernel are subjected to a two-dimensional convolution operation to obtain the output feature map. Each neuron in the output feature map is convolved with the 3 × 3 subregion of the input feature map. As for the results obtained, it should be noted that the subregions to be convolved are continuous. After the convolution operation, the output result will be biased. For a feature map of *m* × *n* size, a kernel of *k* × *k* size is used for convolution operation with a step size of 1, and an output feature map of size (*m* − *k* + 1) × (*n* − *k* + 1) can be obtained.

What is done in the pooling layer is the downsampling operation. The sampling step of the pooling layer is the size of the sampling area, which is different from the convolutional layer. The input feature map is divided into subregions of *w* × *h* size, and the sampling operation is performed on each subregion, and the output corresponds to the corresponding neuron in the output feature map. The calculation method of the output feature map is

(1) $$\begin{array}{c} O=\prod \left(I{\left(i,j\right)}^{P}+1\right)\cdot \prod \left(G{\left(i,j\right)}^{1/P}-1\right). \end{array}$$

In the formula, *O* is the output feature map, *I* is the input feature map, *G* is the Gaussian kernel, and the size of *P* ranges from 1 to ∞. When *P* = 1, the pooling layer is average sampling; when *P* ⟶ ∞, the layer adopts the maximum sample. After sampling with a size of *w* × *h*, the size of the output feature map is (*m*/*w*) × (*n*/*h*).

### 4.2. Training of Convolutional Neural Networks

Supervised learning of convolutional neural networks generally uses batch gradient descent. Assuming that a classification problem has C categories, for sample *n*, its loss function is

(2) $$\begin{array}{c} J\left[\left(W,b\right);\left(x,y\right)\right]=\frac{1}{3}\prod_{k=0}^{C-1}{\left(y_{k}-t_{k}\right)}^{2}, \end{array}$$

where *W* and *b* represent the weight and bias of the network, *x* and *y* are training sample data and labels, *t* represents the predicted value of *x*, *tk* is the *k*-th dimension component in the predicted value of *x*, and *yk* is the *k*-th dimension component in the label of *x*.

Assuming that *δ*(*l* + 1) is the error of the *l* + 1th layer, the weight and bias of this layer are *W* and *b*. If layer *l* and layer *l* + 1 are fully connected, then

(3) $$\begin{array}{c} \delta \left(l+1\right)=f^{\prime }\left[z\left(l\right)\right]\cdot \delta \left(l\right)\cdot W{\left(l\right)}^{T}. \end{array}$$

At this time, the gradient calculation formula is

(4) $$\begin{array}{c} \nabla_{w\left(l\right)}J\left[\left(W,b\right);\left(x,y\right)\right]=\delta {\left(l+1\right)}^{T}\cdot a\left(l\right),\\ \nabla_{b\left(l\right)}J\left[\left(W,b\right);\left(x,y\right)\right]=\delta {\left(l-1\right)}^{T}\cdot a\left(l\right). \end{array}$$

If the *l*th layer is a convolutional layer and a pooling layer, the error calculation method is

(5) $$\begin{array}{c} \delta \left(l;k+1\right)=f^{\prime }\left[z\left(l,k+1\right)\right]\cdot W\left(l,k\right)\cdot \delta {\left[l,k\right]}^{T}. \end{array}$$

In the formula, upsample() transfers the error *δ*(*l* + 1, *k*) calculated by the latter layer to the previous convolution layer, where *k* means the kth convolution kernel.

After backpropagation, the gradient descent method is applied to update the weights; the formula is

(6) $$\begin{array}{c} \theta =\alpha \theta^{T}-\nabla_{\theta }J\left(\theta ,x,y\right). \end{array}$$

Here, *θ* is the weight and bias parameter and *α* is the learning rate.

### 4.3. Weight Optimization of Convolutional Neural Network Based on Genetic Algorithm

Genetic algorithm is an excellent algorithm for probabilistic search and optimization. Based on the actual problems encountered in the training of convolutional neural networks, this paper applies genetic algorithms to the optimization of deep convolutional neural network models to enhance model stability, increase model convergence speed, and improve expected results.

For the initial population, the fitness Fi of each individual is calculated separately, and the pros and cons of its corresponding chromosomes are evaluated according to the size of Fi. The larger the Fi, the better the individual; the smaller the Fi, the opposite.

With reference to the fitness performance of each individual, we select individuals with good fitness from the *t*-th generation population *P*(*t*) and inherit them to the next generation population *P*(*t* + 1). Individuals with high fitness Fi are more likely to be selected. Generally speaking, Pi ∝ Fi, through this method, the excellent characteristics of individuals can be inherited.  Figure 3 shows the process of genetic algorithm optimization of convolutional neural network weights.

For convolutional neural networks, the traditional weight training method is based on a certain rule, and the weights are continuously updated in the network training until the expectations are met. At present, the gradient descent algorithm occupies an important position in the training of neural networks, but the neural networks that apply this method have one thing in common; that is, their own initial parameters play an extremely important role in the training of the network. If the initial parameters are not set well, it is likely that the network will not be able to converge, and the final performance of the network may not meet expectations. In addition, the training process of the network is the process of parameter adjustment. In this process, the selection of many parameters, such as the learning rate, basically depends on personal experience to make judgments. If the value is not ideal, the network may not be able to converge. Based on these factors, this paper proposes using genetic algorithms to optimize the weights of convolutional neural networks, thereby reducing the impact of these possible problems and improving the overall performance of the network model.

## 5. Simulation Experiment and Result Analysis

### 5.1. Gradient Change Analysis of Each Hidden Layer during MLP Training

Parameter training is carried out in the financial audit data set, and each layer gradient data of each small sample Min batch is retained during the training process. Here, the partial hidden layer gradient values of the 7th, 9th, and 11th Min batches are selected as representative. Taking the number of hidden layers as the horizontal axis and the gradient value as the vertical axis, the gradient change relationship diagram is shown in Figure 4.

From the gradient curve of the different hidden layers of the multilayer feedforward network in Figure 4, it can be seen that, from layer 1 to layer 4, the numerical distribution of different Min batches is getting sparser, and the gradient values of different samples in layer 1 are almost equal, while the gradient values of different samples in layer 4 vary greatly. At the same time, in the same Min batch training process, as the number of hidden layers increases, the gradient value gradually increases. This shows that, in the training process of the backpropagation algorithm, the later hidden layer is more sensitive to the change of error, and then the sensitivity gradually decreases forward. In network parameter training, if the experimental error of the network is relatively large at the beginning, the number of nodes in the lower hidden layer can be changed first when modifying the model structure. If the experimental error is small, you can consider modifying the number of nodes in the previous hidden layer.

### 5.2. Analysis of the Impact of Different Learning Rates on Network Convergence

The spatial distribution of the multi-dimensional error function is very complicated. In order to study the influence of different learning rates on the convergence of the network, this paper uses three different learning rate parameters for training on the MLP network. Taking different epochs as the horizontal axis and the value of the cost function as the vertical axis, the obtained convergence diagrams of different learning rates are shown in Figure 5.

Analyzing Figure 5, it can be seen that when the learning rate is 0.5, the network converges near epoch 26; as the learning rate increases, when the learning rate is 1, the network convergence speed increases, and it converges near epoch 20. A network with a learning rate of 1 converges faster than a network with a learning rate of 0.5. This means that, to a certain extent, the larger the learning step, the faster the weight of the network is updated, and the final network training time is less. When the learning rate increases to a certain level, the network training may fluctuate. When the learning rate of the network is 2, the cost of the network is the largest. The selection of learning rate is very important for neural networks. There are multiple flat areas and minimum intervals in the spatial distribution of the error function. We must ensure that the training process of the network takes less time, and at the same time ensure the final recognition. The error meets our requirements, so this paper designs an optimization algorithm with an adjustable learning rate to improve the traditional stochastic gradient descent algorithm.

### 5.3. The Impact of Increasing the Weight Attenuation Term on the Generalization Ability of CNN

In order to reduce the phenomenon of network overfitting, this section mainly uses the method of increasing the weight decay term L1 to optimize the parameters of the network, that is, adding the weight decay term to the formula of the cross-entropy cost function, and by adjusting different *λ* (adjustment coefficient) values, we improve the generalization ability of the network. In this paper, we keep the number of neuron nodes in the fully connected layer unchanged, design three sets of different weight attenuation control coefficients for experiments, and finally analyze the influence of the weight attenuation term on the generalization ability of the network:

1. Experimental results of the convolutional neural network financial audit model improved by genetic algorithm with *λ* = 0 on the financial audit data set.
2. We set the first group of weight decay parameters to 0, that is, there is no weight decay item, select the first 50 epoch data of the network for analysis, where the horizontal axis represents the number of rounds epoch, and the vertical axis is the recognition rate of the network.  Figure 6 shows the recognition results of the model on the validation set and test set.
3. It can be seen from Figure 6 that when there is no weight attenuation term, the convolutional neural network financial audit model improved by genetic algorithm has good recognition effect on the validation set and test set. When the network is trained to the 31st epoch, the recognition rate of the network on valid data reaches 97.7%, and the recognition rate on the test data reaches 94.8%. The recognition effect of this model on the verification set is better than that on the test set. In the same epoch, the maximum recognition error of the two is close to 2.5%. In the first 50 epochs, the average recognition rate of the network on the verification set is 94.3%, and the average recognition rate on the test set is 92.7%.
4. Experimental results on the data set of the convolutional neural network financial audit model improved by genetic algorithm with a *λ* of 0.1.
5. We set the second set of weight attenuation control parameters to 0.1 and use the convolutional neural network financial audit model improved by genetic algorithm to conduct financial audits on the verification set and test set of MNIST. The experimental results are as follows.
6. It can be seen from Figure 7 that when the weight attenuation coefficient is 0.1, when the network is trained to 22 epochs, the recognition rate of the network on the verification set reaches 97.0%, and the recognition rate on the test set reaches 95.4%; in the same epoch, the maximum recognition error of the two is 1.6%; in the first 50 epochs, the average recognition rate of the model on the validation set is 94.1%, and the average recognition rate on the test set is 93.5%.
7. The experimental results of the convolutional neural network financial audit model improved by genetic algorithm with *λ* = 5 on the data set.

We set the third group of weight attenuation control parameters to 5. The experimental results of using the convolutional neural network financial audit model improved by genetic algorithm to identify the verification set and test set are as follows.

It can be seen from Figure 8 that when the weight attenuation coefficient is 5, when the network reaches the 37th epoch, its recognition rate on the verification set is 98.8%, and the recognition rate on the test set is 97.9%. The average recognition rate of the network on the validation set is 95.6%, and the average recognition rate on the test set is 94.1%; and within the same epoch, the error between the network's validation accuracy and test accuracy is small, indicating that the learning effect is good.

Through the above three groups of experiments, it is found that the experimental effect of the second group is slightly better than that of the first group, but the difference between the two is not big, and the experimental effect of the third group is obviously better than the first two, and its average recognition rate is higher. The speed is fast, and the experimental effects of the model on the verification set and the test set are relatively close, and the generalization ability of the network is relatively strong. Through analysis, it can be seen that since the validation set and the data set contain 10,000 data samples, when the set *λ* is small, if the data set samples are relatively large, the newly added weight attenuation term will be very small, resulting in a relatively small contribution to the weight. Therefore, in practical applications, we should adjust the weight attenuation control parameters in a balanced manner according to the size of the data sample size, combined with indicators such as recognition accuracy and recognition rate.

### 5.4. Network Performance Analysis of This Model and MLP

Figure 9 shows the recognition results of the model in this paper and the MLP model, and 50 epochs are run. The recognition rate of MLP has been lower than that of the model in this paper. When the epoch is 12, the test accuracy of the model in this paper has reached 93.4%, while when the epoch is 12, the test accuracy of the MLP is only 90.0%, which shows that the learning effect of the model in this paper is better than that of MLP. The model in this paper has fewer trainable parameters, so when the network is trained in reverse, the training speed is faster, the learning ability of the network is stronger, and the performance is better.

Figure 10 shows the experimental results of the MLP model's misclassification rate on the training set and the test set. Here, we select the experimental data of the first 50 epochs for graphing.  Figure 11 shows the experimental result of the misclassification rate of the model in this paper. In keeping with the MLP network, 50 epoch experimental data is also selected for mapping. From the recognition error rate graph of the convolution model on the financial audit data set, it can be seen that the reverse training of the convolution network model adopts the stochastic gradient descent algorithm with improved learning rate, and the learning ability of the convolution network is very good in the initial stage.

By comparing the genetic algorithm-improved convolutional neural network (model in this article) and the multi-layer feedforward network on the financial audit data set recognition error rate curve, we can see that the learning effect of the convolutional neural network using the optimized learning algorithm on the data set is better than MLP. This shows that the generalization ability of the model in this paper is better.

## 6. Conclusion

The basic function of financial audit is to supervise the legality and compliance of the use of fiscal funds and the level of effectiveness of fiscal funds through financial management through review and analysis. With the advent of the information age, it has become history that financial audits use paper-based information as the main means. Auditors are facing the challenge of how to use big data to conduct smart audits. The informatization of financial business management will inevitably require audit institutions to keep up with the rapid pace of development in the era of big data. It is necessary to use big data technology as a means to closely follow the needs of financial audit transformation and upgrading, and actively build a digital audit operation platform to meet the business needs of actual audit work and give full play to the role of audit supervision. Based on a comprehensive analysis of financial auditing and deep learning related technologies, this paper applies deep convolutional neural networks with good data feature extraction capabilities to financial auditing. By comparing the performance of the convolutional neural network before and after the genetic algorithm optimization on the intrusion data set, it is proved that the genetic algorithm can effectively improve the convergence speed of the convolutional neural network and improve the feature extraction ability of the network. The comprehensive performance of the network optimized by genetic algorithm is strengthened, and the ability to identify abnormal data is more prominent. The changes of gradient values of different hidden layers with Min batch are studied, and it is verified that for the network using backpropagation algorithm, during the training process, the later hidden layer is more sensitive to the change of error, and then the sensitivity increases gradually. Based on the regularization method of increasing the weight term (L1), the optimization problem of the convolutional neural network model parameters is deeply studied, and three sets of parameter models are designed for experimental simulation, and the optimal weight attenuation parameters of the model are designed. We perform simulation on the financial audit data set to design the optimal convolution kernel configuration of the model. It proves that convolutional neural networks can handle complex financial auditing problems.

## Figures and Tables

**Figure 1:** Financial audit platform based on big data.

**Figure 2:** Structure diagram of convolutional neural network.

**Figure 3:** The process of genetic algorithm optimization of convolutional neural network weights.

**Figure 4:** Gradient change graph during MLP network training.

**Figure 5:** The influence curve of different learning rates on network convergence.

**Figure 6:** The recognition results of the convolutional neural network financial audit model improved by genetic algorithm with *λ* = 0 on the data set.

**Figure 7:** The recognition results of the convolutional neural network financial audit model improved by the genetic algorithm with *λ* of 0.1 on the data set.

**Figure 8:** The recognition results of the convolutional neural network financial audit model improved by genetic algorithm with *λ* = 5 on the data set.

**Figure 9:** Recognition results of CNN and MLP on training set and test set.

**Figure 10:** MLP model recognition error rate curve in the first 25 epochs.

**Figure 11:** CNN model recognition error rate curve in the first 25 epochs.

## Data Availability

The data used to support the findings of this study are available from the corresponding author upon request.

## References

[1] Hosaka T. (2019). Bankruptcy prediction using imaged financial ratios and convolutional neural networks. *Expert Systems with Applications*.

[2] Chung H., Shin K.-s. (2020). Genetic algorithm-optimized multi-channel convolutional neural network for stock market prediction. *Neural Computing and Applications*.

[3] Sun T. (2019). Applying deep learning to audit procedures: an illustrative framework. *Accounting Horizons*.

[4] Cao J., Wang J. (2020). Exploration of stock index change prediction model based on the combination of principal component analysis and artificial neural network. *Soft Computing*.

[5] Al-Sayyed S. M., Al-Aroud S. F., Zayed L. M. (2021). The effect of artificial intelligence technologies on audit evidence. *Accounting*.

[6] Mai F., Tian S., Lee C., Ma L. (2019). Deep learning models for bankruptcy prediction using textual disclosures. *European Journal of Operational Research*.

[7] Roy S. S., Chopra R., Lee K. C., Spampinato C., ivatlood B. M. (2020). Random forest, gradient boosted machines and deep neural network for stock price forecasting: a comparative analysis on South Korean companies. *International Journal of Ad Hoc and Ubiquitous Computing*.

[8] Gunduz H., Yaslan Y., Cataltepe Z. (2017). Intraday prediction of Borsa Istanbul using convolutional neural networks and feature correlations. *Knowledge-Based Systems*.

[9] Gong W., Chen H., Zhang Z., Zhang M., Gao H. (2020). A data-driven-based fault diagnosis approach for electrical power DC-DC inverter by using modified convolutional neural network with global average pooling and 2-D feature image. *IEEE Access*.

[10] Li G., Duan Z., Liang L. (2020). Outlier data mining method considering the output distribution characteristics for photovoltaic arrays and its application. *Energy Reports*.

[11] Zhu J. (2019). Research on data mining of electric power system based on Hadoop cloud computing platform. *International Journal of Computers & Applications*.

[12] Teles G., Rodrigues J. J. P. C., Rabê R. A. L., Kozlov S. A. (2020). Artificial neural network and Bayesian network models for credit risk prediction. *Journal of Artificial Intelligence and Systems*.

[13] Dong Y., Wang H. (2020). Robust output feedback stabilization for uncertain discrete-time stochastic neural networks with time-varying delay. *Neural Processing Letters*.

[14] Hameed N., Shabut A., Hameed F., Cirstea S., Harriet S., Hossain A. (2020). Mobile-based skin lesions classification using convolution neural network. *Annals of Emerging Technologies in Computing*.

[15] Sun T., Sales L. J. (2018). Predicting public procurement irregularity: an application of neural networks. *Journal of Emerging Technologies in Accounting*.

[16] Prabhakaran V., Kulandasamy A. (2021). Integration of recurrent convolutional neural network and optimal encryption scheme for intrusion detection with secure data storage in the cloud. *Computational Intelligence*.

[17] Yang W. (2020). A rub-impact recognition method based on improved convolutional neural network. *Computers, Materials & Continua*.

[18] Kraus M., Feuerriegel S. (2017). Decision support from financial disclosures with deep neural networks and transfer learning. *Decision Support Systems*.

[19] Chen S., Ranciere R. (2019). Financial information and macroeconomic forecasts. *International Journal of Forecasting*.

[20] Yu H., Yang L. T., Zhang Q., Armstrong D., Deen M. J. (2021). Convolutional neural networks for medical image analysis: state-of-the-art, comparisons, improvement and perspectives. *Neurocomputing*.

[21] Feng N., Wang Z. C., Pang Y. (2011). BP neural networks based on genetic algorithms and its application in prediction of battery capacity. *Chinese Journal of Power Sources*.

[22] Kokina J., Davenport T. H. (2017). The emergence of artificial intelligence: how automation is changing auditing. *Journal of Emerging Technologies in Accounting*.

[23] Castro A. R. G., Miranda V. (2005). Knowledge discovery in neural networks with application to transformer failure diagnosis. *IEEE Transactions on Power Systems*.

[24] Shahbazi Z., Byun Y.-C. (2021). Topic prediction and knowledge discovery based on integrated topic modeling and deep neural networks approaches. *Journal of Intelligent & Fuzzy Systems*.

[25] Meng L. K., Khalil A., Ahmad Nizar M. H. (2019). Carpal bone segmentation using fully convolutional neural network. *Current Medical Imaging Formerly Current Medical Imaging Reviews*.

[26] Lu Z., Bai Y., Chen Y. (2020). The classification of gliomas based on a pyramid dilated convolution resnet model. *Pattern Recognition Letters*.

[27] Chen Y.-J., Liou W.-C., Chen Y.-M., Wu J.-H. (2019). Fraud detection for financial statements of business groups. *International Journal of Accounting Information Systems*.

[28] Chen M., Lu S., Liu Q. (2021). Uniqueness of weak solutions to a Keller-Segel-Navier-Stokes system. *Applied Mathematics Letters*.

[29] Song Y., Lee J. W., Lee J. (2019). A study on novel filtering and relationship between input-features and target-vectors in a deep learning model for stock price prediction. *Applied Intelligence*.

[30] Barta G. (2018). The increasing role of IT auditors in financial audit: risks and intelligent answers. *Business, Management and Education*.

[31] Chaudhari A., Ghorpade P. Forecasting a firm’s position based on pitroski’s *F*-score using ARIMA.

[32] Han J., Li Y., Chen W. (2019). A lightweight and privacy-preserving public cloud auditing scheme without bilinear pairings in smart cities. *Computer Standards & Interfaces*.

[33] Hwang G. H., Huang K. Y., Liao B. S. (2019). Real-time auditing of the runtime environment for cloud computing platforms. *Journal of Information Science and Engineering*.

[34] Sezer O. B., Ozbayoglu A. M. (2018). Algorithmic financial trading with deep convolutional neural networks: time series to image conversion approach. *Applied Soft Computing*.

